# Machine-Vision-Based Enhanced Deep Genetic Algorithm for Robot Action Analysis

This article has been retracted.

**DOI:** 10.1155/2022/4047826

**Published:** 2022-09-30

**Authors:** Guifeng Wang, Lu-ming Zhang, Yichuan Sheng

**Affiliations:** ^1^Key Laboratory of Crop Harvesting Equipment Technology of Zhejiang Province, Jinhua Polytechnic, Jinhua 321007, Zhejiang, China; ^2^Hithink RoyalFlush Information Network Co., Ltd., Hangzhou, China

## Abstract

The machine-driven products processed by CNC machine tools are divided into multiple parts, which are often transmitted to unqualified processing crystals due to the error of the part's posture, thus affecting the projection effect. Aiming at handling this problem, we, in this work, propose a method for locating and correcting machine capabilities based on bicycle visual recognition. The robot obtains coordinates and offset points through the vision system. In order to satisfy the requirement of fast sorting of the robot parts, a robot species method (BAS-GA) that supports machine vision and improved genetic algorithm rules is proposed. The rank method first preprocesses the part copies, then uses the Sift feature twin similarity notification algorithm to filter the part idols, and finally uses in-law deformation to place the target parts. Afterward, an particular model is built for the maintenance of the nurtural skill, and the mathematical mold is solved using the BAS-GA algorithmic program authority. The close trail of the robot is maintained to manifest the marijuana of the robot. Experimental inference have shown that the BAS-GA algorithm rule achieves the optimal conclusion similar to the pseudo-annealing algorithmic program plant. Meanwhile, the genetic algorithm rule is modified ant settlement algorithm program. Knife sharpening was also reduced by 7%, inferring that this process can effectively improve the robot's action success rate.

## 1. Introduction

Part sorting is a very important link in the industrial production process. The traditional manual sorting is not only inefficient but also time-consuming and labor-intensive and can no longer meet the needs of modern production. At present, some enterprises have applied industrial robots in sorting operations, but their sorting methods are single and cannot adapt to complex scenarios. Machine ken technology has the characteristics of automation, non-contactor, and violent preciseness. Applying coach vision to the sorting process of business robots can thoroughly improve the embroidery efficiency. Gang et al. [1] proposed a method based on the Surf and Freak algorithm.

After decades of development, CNC machining technology has gradually developed from simple part processing with low quality and efficiency to higher processing quality and faster processing efficiency. The product categories are also more abundant, and the traditional CNC machine tools can no longer meet the demand and are gradually eliminated. In the automatic machine tool production line, the market has always had high requirements for the quality and efficiency of processed products, and the quality of machine tool processed products is easily affected. If the machining process is still executed according to the set program, there will be machining deviation, which will cause quality and efficiency problems. The development of CNC machine tools urgently needs to solve this problem. With the rapid development of computer, image processing and recognition technology, machine vision technology is becoming more and more popular and its application is more and more extensive. The current application of machine vision technology mainly covers industry, agriculture, and shipbuilding, for example, product size measurement, appearance defect quality inspection [1], finished product qualification inspection, automatic welding, and other fields. In addition, in the fruit screening system, apple picking system and the use of monocular is proposed.

The optic thesis technology [2] is also complex. Therefore, the coalition of dress vision in the industrial response and the numerical guide machine tools that need to be resolve urgently has become a fiery spot. In the elapsed confederated application of eyeshot and CNC dress puppet, it is mostly reflected in the aspects of machine drive machining weapon, axis situation, and machining projection feature optimization, and the execution is general. The component sorting method, the algorithm speeds up the establishment of the model and reduces the time of target classification. A workpiece sorting system for different shapes, mainly using template matching to classify and locate workpieces. The system can classify workpieces in any position. Wu et al. [3] proposed an algorithm for workpiece recognition based on deep learning, which has good feasibility. The above robotlike species method based on machine eyesight has greatly amended the speed and effectiveness vie with manual sorting but does not revolve optimizing the sorting track to further disapprove the sorting system. Path planning problems such as parts sorting [1] and UAV queue adjustment [4] can be reduced to the travel sales problem (TSP), which is a classic combinatorial optimization problem. It can be described as the shortest path for a businessman to go to several cities, and each city can only pass through once and finally return to the starting point city. At present, many scholars have studied the TSP solution algorithm. Therefore, this kind of algorithm mostly adopts the method of combining several algorithms or improving the operator of the original algorithm. Based on the brainstorming (BSO) algorithm, WuC et al. designed a new type of crossover operator to solve TSP. The algorithm has high accuracy and is not easy to fall into local optimum. Wenzhuang et al. [5] designed an improved ant colony (PSO-ACO) algorithm to solve TSP. The algorithm uses the particle swarm algorithm to cross and mutate the better solution generated by the ant colony algorithm to obtain a better population, but the algorithm is slow in solving in practical application. Probability strategies and genetic operators into the particle swarm optimization algorithm, designed a hybrid particle swarm optimization algorithm (IHPSO), and applied it to solve TSP with high convergence accuracy. Jiang et al. [6] proposed the beetle antennae search algorithm (BAS) in 2018. The algorithm is simple in principle, less computationally expensive, and faster to solve. However, BAS is currently used to solve TSP problems. Based on the above analysis, the TSP problem can be effectively solved by improving the operators of the intelligent optimization algorithm. However, the above algorithms have defects such as high algorithm complexity and slow solution speed. The heuristic mutation operator of the algorithm solves the TSP and is applied to the automatic sorting of parts, which improves the speed of the planning path and shortens the length of the trajectory of the robot arm.

Therefore, a system that combines machine vision and robots is proposed for CNC machine tool processing. This system can effectively improve the accuracy of part identification and positioning and speed up the time it takes for robots to identify and grab parts to CNC machine tools. It is a good method for some small and medium-sized enterprises to improve production efficiency, and the development cost is low, and it is not easy to be constrained by environmental conditions.

Optical positioning techniques [2] are also involved. Therefore, the machine vision group in the industrial room and the CNC bicycle tools that need to be cleaned up have become hot spots. In the joint application of the above-mentioned phantom and CNC machine tool bowl, it is mostly reflected in the aspects of machine tool instrument processing tools, axis position, processing technology feature optimization, etc., and the implementation is general. In a componentized way, the algorithm program speeds up the establishment of the model and overcomes the cluttered time. Jiaji et al. [1] designed a workpiece positioning system to differentiate preparations, mainly wear pattern replication, to classify and place workpieces. The system can classify artifacts in any pose. Wu et al. [3] proposed a kind of artifact notification algorithm rule based on mysterious science, which is practical. The above eye-based automatic rifle method is a good correction for the speed and capability gained by manual sorting but does not estimate the optimization of the troops' field of view to further rectify the sorting system. Path equipment problems such as part sorting [1] and drone pigtail suits [4] can be reduced to a mobile sales problem (TSP), which is a pure combinatorial optimization proposition. It can be said that a businessman walks the shortest trail in several cities, each city can only pass once, and finally returns to the starting point of the metropolis. At present, many scholars have elaborated the TSP interrupt algorithm rules in detail. Therefore, this kind of friendly algorithm program mostly adopts the way of several algorithms that are consistent with or improve the operators of the original algorithm rules. Based on brainstorming (BSO) algorithm rules, Wu et al. used a modern type of crossover operator to solve TSP. The algorithm has complete accuracy and is not suitable for getting caught in an epic optimum. Wenzhuang et al. [5] specify the modified ant colony (PSO-ACO) algorithm to solve TSP. The algorithm program used the prefix-majority algorithm program to cross-change the correct releases produced by the emmet colony algorithm to obtain more populations, but the algorithm was slower to clean up in actual contact. A probabilistic strategy and genetic operator in the group optimization algorithm, designated a hybrid inner bending multiple optimization algorithm rule (IHPSO), and accessed it to solve TSP. High convergence exactness. Jiang et al. [6] In 2018, the annoy-try antenna algorithm program (BAS) was proposed. The algorithmic program beginning is artless, the reckoning amount is slender, and the deliverance success is fast. However, BAS is generally used to solve the TSP proposition. Based on the above analysis, the TSP question can be completely solved by improving the operators of the enlightened optimization algorithm rules. However, the above algorithms have defects such as full entanglement of algorithm programs and agility in later crisis. The heuristic change speculator of the algorithmic program solves the TSP, works on the automatic condition of the ability, corrects the scheduling of the chart channel, and shortens the length of the robot force process.

Therefore, a system combining garment vision and robotics is designed for CNC machining. The system can effectively improve the ability recognition and positioning accuracy, and speed up the robot's recognition of CNC bicycle tools and the measurement of grasping ability. For some niche medium-sized enterprises, improving work ability is a good model, and the development cost is low, and it is not easily bound by environmental requirements.

## 2. Related Work

In 2016, 19 U.S. universities jointly released the Robotics Roadmap: From the Internet to Robots under the auspices of the National Science Foundation. The story predicts that robots will become a new technology that will revolutionize humanity. In the future, robots will be used in every corner of human society. At present, robots are the crystallization of traditional disciplines such as mechanics, material knowledge, machine-like control, sensors, and machinery. In the future, robots will integrate review results in new review areas such as judgment technology, intelligent control, human-computer interaction, data processing, and bionic automation materials, robots will move from unwritten commercial industries to wider application fields such as physics, family, and individuals. According to the statistics of some research directions disclosed in the typical journals in the field of robotics, intelligent supervision, human-computer interaction and sensing technology are the fields that have achieved the most results. The passable phase is the movement of the unwritten robot to the passing phase of the future-aware robot. Compared with traditional robots, new technologies such as restraint, sensory fusion, and human-robot interaction make robots easier to use, safer, and more humane. More progress will be made in this area. At present, although robots have been widely used in various business fields, they mainly complete multiple deterministic tasks in a structured environment. As the requirements for recurrence increase and the narrative field matures, collaborative robots emerge as the times require. Collaborative robots are a product of previous integrated research emerging in artificial intelligence processing. Collaborative robots have certain foreign perception capabilities and humanized operation methods.

In contrast to the unwritten dress usage, this CNC styling weapon supports the integration of dress vision and movement supervision systems and mainly explains the proposition of the production performance and effectiveness of the dressing tool. The CNC processing system supported by clothing visual projection mainly has four systems, namely the shape eye system, the robot system, the motion control system and the CNC system. Among them, the machine vision system has the ability of positioning and projection to identify the position and orientation of interest. The robot system will grab the ability according to the coordinate advertisement fed back by the perception system, and then the CNC system will process the ability. In the work prominence of these three systems, the proposed control systems all need principles and controls to complete the intelligent exchange of each system. In Brie, the operation of CNC machining under the automatic performance linen is described as mimicking: trimming tool machining changes from keyboard transport and food to automatic machine-style seat belt dipping food, the machining capability is immediately sent to the trainer tool food position, and then the robot is used to grab parts and feed them. The machine tool used under the growth of the whole set of automated synthetic ropes reduced the labor. At the same time, for the growth and the white-eye effect, a machine model was added to the feeding position of the car bowl, and the parts grasped by the robot were carefully positioned to remind the robot to understand the assertion. Suitable. Machine phantoms are interested in identifying and locating mucositis of parts. When the part reaches the indicated position and gets in the way, the vision camera runs and unfolds the coordinates of the part through the software. After the robot obtains the non-additional information of the part through the motion rule system, it grasps the part. Take the part and place it in the selected location of the trim tool. At the same time, due to the transit acceleration of the belt line, it may cause the part to tilt when it reaches the food position of the shape tool. After the robot grabs it and absolutely preys on it into the shape instrument, the part also has to be tilted. G-codes for shape puppets have always been literal. Once the part is tilted, it must be a substandard product after bulging, so bulging also requires precise positioning of the curved part to ensure that the part is overbearing when entering the selected position of the machine tool. Machine recognition then also needs to identify the impact scheme of the part and send the angular luminosity to the robot. After the robot grabs the inclined part, it will perform viewpoint correction to ensure the process of the part under the positive guidance and ensure the processing quality. Based on this prominence, there is also a need to push for ubiquitous direct government design to guarantee the proper functioning of automatic performance boundaries and voice enlightenment.

## 3. Our Proposed Method

The system can be simplified as a remote-operated robotic weapon system, and the remote-operated technology uses robotic arms to replace speculators to complete various operations. The key to the remote control robotic arm system is to project the objective behavior of topic speculators onto the robotic arm through the remote control system, so it is necessary to collect speculators' movement data in real time to make decisions. Coincidentally, the research directions of human arm motion data collection are seriously divided into two categories: electronic computer phantom technology devices based on optical sensors and wearable devices based on inertial sensors. These two methods have their own advantages and disadvantages, but the method supported by the inertial sensor is more suitable and practical in the case where the touch environment of the optical sensor is tense.

Due to the advancement of microelectronics technology, the integration of MEMS devices is getting higher and higher, and the inertial sensors with complex sources are getting smaller and smaller. Therefore, MEMS inertial sensors have wider and more flexible applications due to their cheap and compact characteristics. The data acquisition device proposed in the iron part of the wearable human body mainly uses the MEMS inertial sensor to measure the amplitude and attitude of the soil block, and then cleans the movement data of the soil block. The system uses MPU9250 as an merged inertial mensuration dress, including a three-arbor accelerometer, a three-cross gyroscope and a three-spotted deer magnetometer. The accelerometer and magnetometer in the MPU9250 have a severe cry, so the instantaneous values of the accelerometer and magnetometer's production foreshadowing are not critical enough, and the pose that immediately fits will wobble, but the long-term data of the accelerometer and magnetometer are durable. On the other hand, the gyroscope has low noise, i.e., the raw velocity obtained in each result is relatively accurate, but due to the use of integrals to estimate the rotation angle there will be a component aggregate drift, the inaccuracy of the repine-term data gyroscope, i.e., the gyroscope foreground Phenomenon. Based on the complementary properties of the accelerometer, magnetometer, and gyroscope in the crowd domain, these three sensor data can be fused to correct the system's realism and operational characteristics. When the MPU9250 is stationary, theoretically, the viewpoint limited by the reduced size of the accelerometer/magnetometer *XYZ* is projected into the 3D coordinate system. The inner core of the sphere is an ellipsoid at the origin, but the perfect inner core is offset from the origin due to sensory craft errors. The ball reporter finds the branch at the center of the ball. The appropriate problem for the ellipsoid is to solve the pivot axis of the ellipsoid according to the coordinate step size, abbreviated as the following array form:

(1) $$\begin{array}{c} X=\left(\text{KT }K\right)-1, \end{array}$$

where *x*, *y*, and *z* means the weights, respectively.

Do not actually measure the *XYZ* axes of an accelerometer or magnetometer. By expanding the above matrix equation with the minimum level process, the characteristic matrix can be solved, and the spherical core coordinates can be solved according to the characteristic matrix. The base coordinate system of the magnetometer and the base coordinate system of the accelerometer are different, so the magnetometer coordinate system must be converted to the accelerometer coordinate system. Assuming that the gravitational acceleration measured by the accelerometer is ag, and the magnet variable vector uniformly obtained by the magnetometer is *Φb*, first convert the unnamed coordinates of the magnetometer into the base coordinates of the accelerometer, that is, *Φa* = *AΦb*, A is the rotation, and the ellipsoid is regenerated to become a dogmatic sphere spreadsheet.

After the recognition and attitude of the nut parts are supplemented, the manipulator's path planning ability for the nut is stimulated. Let it be the adjustment of the movement sequence and the “target part”, and 100 million be the good path of the manipulator under this poor run:

(2) $$\begin{array}{c} \text{Heart}=\text{Tune}/\left({}^{“};,{}^{”}+1\right). \end{array}$$

Among them: *d*(%, % + *d* is the “part”; the coldness is the part of the island. It can be seen that the model has a reputation for the TSP problem.

A genetic algorithm (GA) is an anapophysis that mock biologic maneuver. According to the term of outliving of the fittest, optimal destruction is finished through population maneuvers. The breach projection of the GA program playbill is as follows. First, each target part is encoded, and the sequence of each digest in the gene arrangement is taken as a separate, that is, a robotic sorting path. After the encoding is complete, a population with qualified adjustments is randomly generated, which can be converted into a set of paths of different ranks. The fitness responsibility plays an important role in optimization advancement. In the manipulator classpath optimization process, the goal of the troop path is to be the shortest. The fitness function is defined in the following.

After determining the fitness service, wake up the population to perform various trading operations such as quotation, crossover, and change; calculate the fitness of each individual; and obtain the feature with the highest fitness, that is, the optimal path of the robot class. A change operation is a random change in the genetic posture of individuals in a population. Common mutation trading operations include cross mutation, reverse mutation, and switch mutation.

The beetle search algorithm (BAS) is an improved algorithm rule based on the foraging principle of scarabs. The repine dorbeetle has two tentacles. When lingering scarabs are foraging, the two antennae sense the main nutritive odor. If the concentration of taste judgments by the right antennae is greater than that of port one, it will move to the right antennae, and vice versa. The beetle search algorithm has the characteristics of high global detection success rate and high release accuracy, and has been widely used in changing industrial fields. As described above, the abolition change of the GA algorithm program is to change the evaluation of some genes of the individuals in the population, with indisputable credibility, with rich randomness, and plunge into the fitness of poverty, which focuses on the algorithm program capabilities and expeditions.. To correct the algorithm's ability, a heuristic mutation speculator is designed to fit the problem of this paper and the fantasy of the BAS algorithm program. That is, in each transform fold, only the nearest boundary tattered part can be selected as the next position. Protrusions are represented by causes as A = black magic, i.e., conditional sidewalks. Unused specific spawns are represented as dangerous choices from the parent A to select the target part, which is represented as a, which is the starting stage of B. The two sides of the part is the monument as 5, the coolness between the ability and a is d^drO. Here, a can be understood as the incidental attitude of the clock and the answering worm's left and right whiskers, feeling and heart. Corresponding to the smell of the left and right whiskers, by comparing the odor intensity on both sides, the next position of the beetle is firm. Adding the obtained proposition to B, in order to verify the validity of the discourse speculator, and using the international standard TSPUB test data to try burst4, the known ideal solution of burst4 is 30.87, and the modified mutation can be proficiently obtained to improve the fitness, so as to find the best release at a faster speed.

## 4. Experimental Results and Analysis

In the system that confirms the rule performance of the BAS-GA algorithm, the data Ulysses22, att48, and eillO1 in TSPLIB are selected for feint experiments. The above data are the city coordinates of the example of the travel anti-jumper proposition, which is mainly used to test the performance of TSP related algorithms. In this paper, different algorithms are used for comparative experiments. To guarantee the fairness of the proof, all experiments are captured in the same environment. The specified simulation environment is as follows: the working (predicate) system is Windows 10, the CPU model is AMD 3100, and the working (predicate) environment is Matlab2020a. In the BAS-GA algorithm, the population size is 100, the crossover cost is 0.3, the change proportion is 0.7, and the enumerate of iterations is circumscribed to 500. Algorithm (GA) and Improved Emmett Settlement Algorithm (PSO-ACO) in Letters [5]. We present the most solution ex cathedra announced by Opt Entertainment, Best show the largest seen length obtained experimentally, and time relate the cadency of obtaining an intellectual also. In order to make the existing data more suitable, this paper uses the relative error Er to evaluate the interrupt correctness of the algorithm, which is the evaluation obtained by multiplying the ratio of the absolute error to the correct value by 100%. As can be seen, GA algorithm program and PSO-ACO algorithm rules.

The BAS-GA algorithm has higher solution accuracy and shorter transfer metrics. At the same time, for the data of Ulysses22, the BAS-GA algorithm looks for a shorter path than the official data. However, from the data set eill01, the BAS-GA algorithm program may change to save the best when determining transactions with a large amount of data. Compared with the PSO-ACO algorithm, although the BAS-GA algorithm leads in solving age, it has The granularity of the loose is illustrious, but it lags in the justness of the crisis and necessarily to be kept timely. After inputting the center coordinates of the nut capability into the pairing device, customize the opening path and honing path to control the grasping of the manipulator, and read out the coils of the manipulator route under the two paths.

The system framed an unassembled optical propulsion podium through the Sketch Vision system and designed a UI manifest interface for counterfeiting analysis, which can clearly display the learned data advertisement, such as the bit of projection ability attitude coordinates and offset steering. It is quiet about necessity and very scalable. An example of non-composite recognition is a utility for distinguishing between activities performed by a system. First, create the banner template and identify the follow-up section and use this status as a color for secondhand. In this tense, the coordinates and angles of the part are *X* = 397.00, *Y* = 401, and *R* = 0.00, respectively. After the speed proposition ability is invested, the spring that distinguishes the position *X*, *Y* and the plan attack, *X* = 408.00, *Y* = 381.00, *R* = 26.98. After being saved by the system, the *X*, *Y* position information is transmitted to the manipulator through the heading control, and the deviation angle is transmitted to the rotation servo model. The robot grabs the *X* and *Y* positions and rotates and penalizes the inflection point map *R* by rotating the servo model to keep the project dogmatic, i.e., consistent with the logo template map. The positioning section has an insidious deflection angle of 26.98°. After remediation, it is rotated 27° to the right, and the fallacy is only 0.02°. The rise of restoration schemes is shown in the following. The system first proposes a CNC machining scenario through practical simulation software and tests it in the actual environment. Simplify the process of simulating machine tool protrusion orientation with a trainer vision and gesture guidance system. The cool image is first captured by the camera in the simulation software, and then the captured actors are put into the processing system for monochrome processing. Then, the similar median filtering behavior is realized, which eliminates the disturbing cry and greatly improves the color filtering effect. Then, the image is hinged through the base value to destroy the useless area, and the docking object is obtained, which is convenient for processing. Then, the essence of incite is to identify the set state of the slice, calculate the complete moment feature to obtain the deflection and coordinates, and convert the coordinate system of the robot through the calibration algorithm program. Floor-planning and routing of guard lines. Ultimately, machine vision and direct inspection systems in physical and virtual production lines can be carefully identified, located, and universally operated.

Before adopting the vision system, the joint propulsion test used by the robot and the trainer was inclined, and the machining parameters without perception guidance were successful, and the machining parameters of the same part under the eye diagram system were obtained. At present, the system has been applied to external small tabletop crockery. The Hikvision camera is the conceptual acquisition and image processing part of the habitual realization of the eye system. The Kaibao robot is used to accept the attitude suggestion sent by the phantom system to achieve part positioning, capture, and tangent punishment. Parts sent by the open-type pyramid robot of the sculpture machine come with the three-axis linkage saver; desktop office generally can meet various processing constraints. In practical application, part recognition, assertion, and wrapping effects are a few examples. The complete product was processed under the guidance of the vision system. The glyptic pattern is centered, and the fruit is qualified. It can be confirmed that under the visible notification effect, after the robot is trained to the perfect deflection ability, the qualified products can become bony protrusions. The reliability of the vision system is then verified.

## 5. Conclusions

In order to improve the automatic sorting efficiency of parts, this paper uses machine vision technology to identify and locate parts, establishes a TSP model for the coordinates of the obtained target parts, and designs a BAS-GA algorithm to solve the model. By comparing the BAS-GA algorithm with a variety of algorithms, the BAS-GA algorithm has a shorter path planning time and higher solution accuracy. The algorithm has good advantages and feasibility and is suitable for practical engineering applications.

## Data Availability

The figures and tables used to support the findings of this study are included in the article. The data can be acquired by requesting the correspondence author.

## References

[1] Haojian Z., Tingting S., Wu S. (2017). Sorting path optimization of parallel robots based on improved genetic algorithm. *Journal of South China University of Technology*.

[2] Liao J., Jianqun L., Gao W. (2019). Design of robotic sorting system based on machine vision. *Combined Machine Tool and Automated Processing Technology*.

[3] Wu X., Guoming H., Lining S. (2016). Fast visual recognition and localization algorithm of industrial sorting robot based on deep learning [J]. *Robot*.

[4] Wei Y., Changjiang L., Shanjun L. (2020). Path planning method for agricultural UAV based on differential quantum annealing algorithm [J]. *Journal of Huazhong Agricultural University*.

[5] Wenzhuang L., Jiayong C., Mingzhang D. (2019). Application of improved ant colony algorithm in welding robot path planning [J]. *Mechanical Design and Research*.

[6] Jiang X. Y., Li S. (2018). BAS: beetle antennae search algorithm for Optimization Problems. *International Journal of Robotics and Control*.

